The article "Recognition of Flexion and Extension Imagery Involving the Right and Left Arms Based on Deep Belief Network and Functional Near-Infrared Spectroscopy" was published in 2021. Journal: J Healthc Eng.

# Recognition of Flexion and Extension Imagery Involving the Right and Left Arms Based on Deep Belief Network and Functional Near-Infrared Spectroscopy

**DOI:** 10.1155/2021/5533565

**Published:** 2021-06-29

**Authors:** Yunfa Fu, Rui Chen, Anmin Gong, Qian Qian, Ning Ding, Wei Zhang, Lei Su, Lei Zhao

**Affiliations:** ^1^Faculty of Information Engineering and Automation, Kunming University of Science and Technology, Kunming 650500, China; ^2^Brain Cognition and Brain-Computer Intelligence Integration Group, Kunming University of Science and Technology, Kunming 650500, China; ^3^Brain Science and Visual Cognition Research Center, School of Medicine, Kunming University of Science and Technology, Kunming 650500, China; ^4^Yunnan Provincial Key Laboratory of Computer Technology Applications, Kunming, China; ^5^School of Information Engineering, Chinese People's Armed Police Force Engineering University, Xian 710000, China; ^6^Kunming Medical University, Kunming 650000, China; ^7^Faculty of Science, Kunming University of Science and Technology, Kunming 650500, China

## Abstract

Brain-computer interaction based on motor imagery (MI) is an important brain-computer interface (BCI). Most methods for MI classification are based on electroencephalogram (EEG), and few studies have investigated signal processing based on MI-Functional Near-Infrared Spectroscopy (fNIRS). In addition, there is a need to improve the classification accuracy for MI fNIRS methods. In this study, a deep belief network (DBN) based on a restricted Boltzmann machine (RBM) was used to classify fNIRS signals of flexion and extension imagery involving the left and right arms. fNIRS signals from 16 channels covering the motor cortex area were recorded for each of 10 subjects executing or imagining flexion and extension involving the left and right arms. Oxygenated hemoglobin (HbO) concentration was used as a feature to train two RBMs that were subsequently stacked with an additional softmax regression output layer to construct DBN. We also explored the DBN model classification accuracy for the test dataset from one subject using training dataset from other subjects. The average DBN classification accuracy for flexion and extension movement and imagery involving the left and right arms was 84.35 ± 3.86% and 78.19 ± 3.73%, respectively. For a given DBN model, better classification results are obtained for test datasets for a given subject when the model is trained using dataset from the same subject than when the model is trained using datasets from other subjects. The results show that the DBN algorithm can effectively identify flexion and extension imagery involving the right and left arms using fNIRS. This study is expected to serve as a reference for constructing online MI-BCI systems based on DBN and fNIRS.

## 1. Introduction

In order to improve the classification accuracy for brain-computer interfaces (BCIs), a deep belief network (DBN) was designed to classify functional near-infrared spectroscopy (fNIRS) signals. This paper used oxygenated hemoglobin (HbO) concentration as a feature to train two restricted Boltzmann machines (RBMs) which were subsequently stacked with an additional softmax regression output layer to construct a DBN. The main goal of BCI is to bypass peripheral nerves and muscles to establish direct communication and control between the brain and the outside world. In addition, this study aims to provide optional communication and control functions for patients with severe motor disabilities to improve their quality of life as well as enhance certain functions for healthy people [1]. fNIRS is an active measurement method in which near-infrared light (650∼1000 nm) is injected into brain tissue by a transmitting probe and collected by a receiving probe. Currently, fNIRS plays a promising role in the clinical area for diagnosis purpose [2–5]. It uses changes in light intensity to calculate oxygenated and deoxygenated hemoglobin concentrations, and functional neurological activity is indirectly inferred from this metabolic activity [6–8].

Motor imagery (MI) is an important paradigm in several types of BCI paradigms [9, 10]. Currently, most methods for MI classification are based on electroencephalogram (EEG), while less attention has been paid to fNIRS. Compared to EEG, fNIRS is a relatively new method for brain imaging and brain-computer interaction [11–13]. One of its advantages is its ability to tolerate a certain degree of movement of the subject's head. In addition, it is highly portable and suitable for monitoring dynamic changes of oxygenation and deoxygenated hemoglobin concentration in brain tissue during movement and imagining; it has also been applied successfully in many fields [14–23]. Studies have shown that MI-BCI based on fNIRS (fNIRS-MI-BCI) is feasible and has several potential applications [24–26].

There is a need to equally improve the classification accuracy of fNIRS. Commonly used classifiers for fNIRS-MI-BCI include support vector machine (SVM) and linear discriminant analysis (LDA). Sitaram et al. used SVM to classify MI tasks and achieved an average classification accuracy of 73.1% [27]. Hoper and Wolf used LDA to classify MI with different time windows, with an average classification accuracy of 81% recorded [28]. Naseer and Hong used LDA to classify tasks at different time windows for an fNIRS signal and achieved an average classification accuracy of 77.5% [29]. However, in these studies, the time window for feature extraction is too far apart from the time point at which the tasks start, and the features are artificially divided, making it difficult to convert them into online systems. Even though deep learning has been successfully applied in several areas [30], it has limited applications in fNIRS-BCI [31–33]. Hennrich et al. first used the deep learning method based on fNIRS to classify different psychological tasks (mental (MA), word generation, and mental rotation (MR)), with a classification accuracy of less than 70% [31]. Therefore, in this paper, we attempt to classify two classes of MI fNIRS signals using the DBN method to verify the validity of the method. The combination of unsupervised and supervised method can improve classification accuracy and training speed. To the best of our knowledge, this is the first attempt at applying the DBN method to MI classification using fNIRS signals.

Deep learning is a descriptively powerful neural network. RBM and automatic encoders are basic modules used in deep learning schemes. They are trained layer by layer [34]. According to the Gibbs Sampling Theory, contrast divergence (CD) is an effective method for training RBMs [35]. Significant improvement in performance can be achieved by initializing multilayer neural networks using features extracted by the RBM in the pretraining phase [36].

In this study, we hypothesized that an RBM-based deep learning method can effectively improve the accuracy of MI classification based on fNIRS. In order to test our hypothesis, fNIRS signals from 16 channels covering the motor cortex area were recorded for each of 10 subjects executing or imagining flexion and extension involving the left and right arms. The DBN algorithm is designed to identify flexion and extension imagery. The optimal parameters and structure settings of DBN were determined by the experiment to generate an optimal classification model.

## 2. Materials and Methods

### 2.1. Subjects

A total of 10 graduate students from Kunming University of Science and Technology were recruited (male, right-handed, with an average age of 24 ± 2 years). All subjects have no movement disorder, and hearing and vision were normal or corrected to normal. Informed consent was signed before the experiment, and the study was approved by the Medical Ethics Committee of Kunming University of Science and Technology.

### 2.2. Experimental Paradigm Design and Experimental Process

The experimental paradigm is shown in Figure 1. The task cue is presented for 2 s, suggesting that, for one of the four types of tasks (left arm flexion and extension execution (L-FE_ME); right arm flexion and extension execution (R-FE_ME); left arm flexion and extension imagery (L-FE_MI); right arm flexion and extension imagery (R-FE_MI)), each task appears randomly. After the cue is removed, the task lasts 8 s and the subject is asked to perform one of the four tasks. During execution of the task, the screen displays the “ ^*∗*^” sign, and the subject is required to keep the head still and avoid blinking. After the task is completed, the test cue is presented for 1 s; the task lasts 17 s; the screen remains blank during the break; the subject can relax and blink normally. The specific experimental procedure is as follows: in a quiet, light-filled room, the test subject is quietly seated 70 cm from a computer screen. The subject's arm is placed flat on a table, with the palm facing down. First, the subject is asked to relax for 3 minutes to calm down. Then, following text prompts on the screen, the subject is asked to perform executed or imagined flexion and extension involving the left and right arms. Each trial comprises 8 s task time and 17 s rest time, as shown in Figure 1(a). During the execution of flexion and extension involving the left and right arms, the subjects are asked to raise the corresponding left or right arm at a speed of about 1 Hz to approximately 90 degrees. During imagery of flexion and extension involving the left and right arms, the subjects were asked to imagine flexion and extension involving the left and right arms in the first perspective. The flexion and extension imagery involving the left and right arms are consistent with those of execution. Flexion and extension movement or imagery involving the left and right arms appear randomly, and the experiment consists of three sessions (30 trials per session) and 90 trials per task. Data from the first two sessions are used as the training set, whereas data from the last session are used as the test set. The fNIRS data obtained from the tasks are analyzed to evaluate the validity of the DBN algorithm.

### 2.3. fNIRS Signal Acquisition

fNIRS signals were collected using a multichannel wireless commercial fNIRS system (NirScan, HuiChuang, China) with a sampling rate of 20 Hz and wavelengths of 740 nm and 808 nm. According to the structure and configuration of the system, six launch probes with eight receive probes were placed in such a way as to cover the motor cortex. The probe layout consists of 16 long-distance channels (30 mm) as shown in Figure 2(a). The experimental setup is shown in Figure 2(b).

### 2.4. fNIRS Data Preprocessing

To eliminate artifacts in the original fNIRS signal, they are bandpass-filtered from 0.01 to 0.2 Hz to eliminate physiological noise caused by heartbeat, respiration, and Mayer waves [37]. The filtered fNIRS signal is then converted to an oxygenated hemoglobin (HbO) signal using supporting data processing software. HbO data for 0∼8 s are extracted after the start of the task and the data for each channel are normalized through linear transformation.

### 2.5. DBN Classification Model

After preprocessing the data, the DBN classification model is trained using the HbO data for flexion and extension movement or imagery involving the right and left arms. DBN is a deep learning method that can be constructed by stacking the autoencoder or RBM. In this paper, RBM was selected for constructing the DBN and the algorithm was implemented using MATLAB 2010a deep learning toolbox. The computer used had the following specifications: i73630QM processor running at 2.4 GHz and 4 GB of memory. The DBN training process comprises two phases: the pretraining phase for each RBM and precise adjustment for the stacked RBM and the softmax regression phase. In the pretraining phase, the input into the RBM is the HbO time series data of flexion and extension movement or imagery involving the right and left arms. Each one-way RBM is individually trained in an unsupervised manner, and pretraining is conducted to reconstruct the input data at the output layer without providing tag information. After fully training the two RBMs, the final DBN is fine-tuned in a directional manner using the conjugate gradient method. The fine-tuning is performed in a supervised manner. The fine-tuning phase can be further divided into two phases: in the first phase, only the weight of the corresponding offset term connected to the output layer is adjusted; the second phase involves the adjustment of all the parameters in the entire network. The obtained parameters can be applied directly to the new input data, thereby enabling efficient data classification.

#### 2.5.1. RBM

RBM is a two-layer (visible layer and hidden layer) neural network that operates in an unsupervised manner [35]. The input data is designed directly as a visible layer and the hidden layer is designed to reconstruct the input data as closely as possible. The visible layer is connected to the hidden layer, and there is no connection between neurons in the same layer. Neurons in the visible and hidden layers are random binary units.  Figure 3 shows a schematic of a single RBM.

The energy function of an RBM is given by

(1) $$\begin{array}{c} E\left(v,h\right)=-\sum_{i=1}^{m}a_{i}v_{i}-\sum_{j=1}^{n}a_{j}h_{j}-\sum_{i=1}^{m}\sum_{j}^{n}v_{i}h_{j}w_{ij}, \end{array}$$

where *v*_*i*_ and *h*_*j*_ represent, respectively, the states of the *i*-th visible unit and the *j*-th hidden unit and *w*_*ij*_ is the connection weight of the *i*-th visible unit and the *j*-th hidden unit. The offset of the visible unit is *a*_*i*_; the offset of the hidden unit is *b*_*j*_.

Based on the definition of RBM energy function, a joint probability distribution for (*v*, *h*) can be obtained as

(2) $$\begin{array}{c} P\left(v,h\right)=\frac{\exp\left(-E\left(v,h\right)\right)}{Z},\\ Z=\sum_{\left(\tilde{v},\tilde{h}\right)}\exp\left(-E\left(\tilde{v},\tilde{h}\right)\right), \end{array}$$

where *Z* is the normalization factor. Though the parameter *W* of the model can be obtained by training, a distribution determined by *W* cannot be calculated accurately. As shown in Figure 3, when the state of the visible cell is given, the activation probability of the hidden unit is conditionally independent. The activation probability of the *j*-th hidden unit is

(3) $$\begin{array}{c} P\left(h_{j}=1|v\right)=\text{sigmoid}\left(v^{T}w_{j}\right)=\frac{1}{1+\text{exp}\left(-v^{T}w_{j}\right)}, \end{array}$$

where *w*_*j*_ denotes the *j*-th column of the connection matrix *W* and the activation of the hidden unit *j* is determined by the inner product (similarity) of the feature *w*_*j*_ of the hidden unit and the input data, *v*. The larger the inner product of the observed data, *v*, and the feature, *w*_*j*_ (the more similar the two vectors), the greater the possibility that the hidden unit *j* is activated. Due to the symmetrical structure of RBM, when the state of the hidden unit is given, the activation probability of the visible unit is also conditionally independent:

(4) $$\begin{array}{c} P\left(v_{i}=1|h\right)=\text{sigmoid}\left(w_{i}h\right)=\frac{1}{1+\exp\left(w_{i}h\right)}, \end{array}$$

where *w*_*i*_ denotes the *i*-th row of the connection matrix, *W*. For observed data *v* in practical problems, how to determine the distribution *P*(*v*) defined by RBM is important. That is, how to determine the edge distribution of the joint probability distribution, *P*(*v*, *h*). It is a product of the experts' model:

(5) $$\begin{array}{c} P\left(v\right)=\frac{\prod_{j}\left(1+\exp\left(v^{T}w_{j}\right)\right)}{Z}. \end{array}$$

It can be seen from equation (5) that each hidden unit contributes a probability to the model according to its similarity with the observed data (*v*^*T*^*w*_*j*_). For observation data, the more the number of features of the hidden unit in the RBM that are similar to the observation data, the higher the likelihood that the observation data are in the RBM.

#### 2.5.2. RBM-Based Learning Algorithm

RBM defines a probability distribution for the observed data, *v*, the parameters of which are obtained by maximizing the log-likelihood of the RBM in the training set; that is,

(6) $$\begin{array}{c} W^{*}=\underset{W}{\arg\max}\sum_{n}\log\;P\left(v^{n};W\right). \end{array}$$

For the training data, *v*(*n*), the gradient of the log-likelihood is given by

(7) $$\begin{array}{c} \frac{\partial \log P\left(v^{\left(n\right)}\right)}{\partial W}=-{\frac{\partial E\left(v^{\left(n\right)},h\right)}{\partial W}}_{p\left(h|v^{\left(n\right)}\right)}+{\frac{\partial E\left(v,h\right)}{\partial W}}_{p\left(v|h\right)}, \end{array}$$

where 〈.〉*P* represents the expectation about the distribution, *P*. As described above, the likelihood of the training data cannot be calculated accurately due to the existence of a normalization factor. Therefore, CD can be used to approximate the logarithm of the log-likelihood (7) of the second term [32]. Specifically, the CD algorithm can obtain a biased estimate of the maximum likelihood solution. To obtain the maximum likelihood solution, the initial training of the RBM can be performed by the CD algorithm, and then, the step size of the Gibbs sampling in the CD algorithm is gradually increased in the subsequent training. A good approximation of the maximum likelihood solution is usually obtained. Therefore, the aforementioned learning rules can also be expressed as optimizing the weight change during RBM:

(8) $$\begin{array}{c} \Delta w_{ij}=\varepsilon \left(v_{i}h_{j\text{ data}}-v_{i}h_{j\text{ recon}}\right), \end{array}$$

where *ε* is the learning rate. Similarly, the learning rules for the deviation terms are

(9) $$\begin{array}{c} \Delta a_{i}=\varepsilon \left(v_{i\text{ data}}-v_{i\text{ recon}}\right),\\ \Delta b_{j}=\varepsilon \left(h_{j\text{ data}}-h_{j\text{ recon}}\right). \end{array}$$

Independent RBMs can be trained by following the learning rules in equations (6), (7), and (8). The pretraining phase of the DBN is described above. It should be noted that each pretrained RBM is intended to reconstruct the input data in the hidden layer and the pretraining phase is performed in an unsupervised manner.

#### 2.5.3. DBN Construction

After separately training two RBMs, the DBN can be constructed by stacking the RBMs one by one. The structure of the DBN is shown in Figure 4. The state vector of the hidden layer in the lower RBM serves as the input to the upper visible layer. The input is fed to the hidden layer of the upper RBM. The state vector of the upper hidden layer serves as the input to softmax regression, whereas the top is the output layer.

As an extension of logistic regression, softmax usually deals with binary classification problems for solving multiple classification problems. Given a training sample, {(*h*_(1)_^*k*^, *y*_(1)_)，(*h*_(2)_^*k*^, *y*_(2)_),…, (*h*_(*M*)_^*k*^, *y*_(*M*)_)}, where *M* is the number of training samples, *k* is the number of iterations, and {(*h*_(1)_^*k*^), (*h*_(2)_^*k*^),…, (*h*_(*M*)_^*k*^)} is the hidden vector of DBN. All parameters of the softmax regression are denoted as *w*, and for *j* = 1, 2,…, *c*, the conditional probability, *P* (*y* = *j*|*h k*), can be written as

(10) $$\begin{array}{c} \left[\begin{array}{c} p\left(y_{\left(i\right)}=1|h_{\left(i\right)};w\right)\\ p\left(y_{\left(i\right)}=2|h_{\left(i\right)};w\right)\\ \vdots \\ p\left(y_{\left(i\right)}=c|h_{\left(i\right)};w\right) \end{array}\right]=\frac{1}{\sum_{j=1}^{c}e^{w_{j}^{T}h_{\left(i\right)}}}\left[\begin{array}{c} e^{w_{1}^{T}h_{\left(i\right)}}\\ e^{w_{2}^{T}h_{\left(i\right)}}\\ \vdots \\ e^{w_{c}^{T}h_{\left(i\right)}} \end{array}\right]. \end{array}$$

The loss function of softmax regression takes a form similar to logistic regression, as shown in equation (11):

(11) $$\begin{array}{c} J\left(w\right)=-\frac{1}{M}\left[\sum_{i=1}^{M}\sum_{j=1}^{c}1\left\{y_{\left(i\right)}=j\right\}\log\;p\left(y_{\left(i\right)}=j|h_{\left(i\right)}^{k};w\right)\right], \end{array}$$

where 1 {·} is the indication function, it has a value of 1 if the input statement is true; otherwise, it is 0. Equation (11) uses the conjugate gradient method to minimize the cost function, and the obtained error term is backpropagated through the multilayer RBM to fine-tune the parameters. The method of fine-tuning the parameters is as described above. Without loss of generality, the updated rules for top-level weights can be written as

(12) $$\begin{array}{c} w_{ij}=\alpha w_{ij}-\varepsilon \nabla_{w_{ij}}J\left(w\right), \end{array}$$

where *α* is the momentum and *ε* is the learning rate. Other layers have similar weight update rules.

In this paper, the DBN is evaluated using the classification accuracy. The number of hidden units in the DBN is determined experimentally. The optimal hidden unit number is selected using the pairwise cross-validation method from the array [10, 20, 30, 40, 50]. In the pretraining phase, the number of RBM training samples is determined experimentally. In this paper, the RBM is stable if the number is greater than 5, so the number of training samples per RBM is set to 10. The learning rate for the weights and deviations is set to 0.1. The momentum is set to 0.5. The HbO concentration data serve as input data to the DBN. One trial per channel consists of 160 data points and 16 channels; the data at each sampling time point are taken as a sample. Therefore, the input data for the RBM are a 16-dimensional vector. For one subject, flexion and extension movement involving the right and left arms or flexion and extension imagery involving the right and left arms include 90 trials. The experiment comprises three sessions (30 trials per session); data from the first two sessions serve as training set, while data from the last session serve as test set. The training set is 19200 × 16, while the test set is 9600 × 16. At the same time, considering differences in classification models trained by individual subjects, this paper also uses test sets from different subjects to evaluate individual differences in the classification models.

## 3. Results

Data obtained from each trial for the 10 subjects were extracted and averaged according to the four defined types of tasks. The average fNIRS response obtained for flexion and extension movement or imagery involving the right and left arms is shown in Figures 5(a) and 5(b). During flexion and extension movement involving the right and left arms, blood oxygen concentration in the brain tissue showed the following trend: the concentration of HbO increased while that of deoxygenated hemoglobin (HbR) decreased, and contralateral motor cortex activation was observed. Flexion and extension imagery involving the right and left arms followed a similar pattern, but the amplitude was weaker. The right side of Figure 5 shows a topographical map of HbO concentration in the motor cortex for the first 8 s after the start of the task, visually showing the difference in activation intensity of the contralateral motor cortex.

The DBN was trained using HbO concentration data during performance of tasks for the 10 subjects. The training set was 19200 × 16, the test set was 9600 × 16, and the number of units in the hidden layer [*h*_1_, *h*_2_] was determined from the array [10, 20, 30, 40, 50] by the cross-validation method.  Table 1 shows the DBN classification accuracy for flexion and extension movement or imagery involving the right and left arms. For flexion and extension movement involving the right and left arms, the average classification accuracy was 84.35 ± 3.86%; the highest classification accuracy recorded was 89.21%, while the lowest classification accuracy achieved was 76.23%. For flexion and extension imagery involving the right and left arms, the average classification accuracy was 78.19 ± 3.73%; the highest classification accuracy recorded was 82.93%, while the lowest classification accuracy achieved was 73.96%.

Additionally, to compare the differences, generalization, or transfer between DBN models trained using different training sets, MI data of the third session for each subject were used as test set to evaluate DBN models trained with each subject. The classification results are shown in Table 2. For the DBN classification model, better classification results were achieved for the test set for a particular subject when the DBN model is trained with training set from the same subject than for test sets in which the same DBN model was trained with training set from other subjects.

## 4. Discussion

In this paper, we explored the feasibility of the recognition of flexion and extension movement or imagery involving the right and left arms using DBN and fNIRS. The proposed method achieves a higher classification accuracy (78.19 ± 3.73%) for two types of MI fNIRS signals based on DBN compared to the traditional algorithms adopted by Sitaram et al. [27], Naseer and Hong [29], and Zhang et al. [38] (average classification accuracy: 73.1%, 77.5%, and 75.3%, resp.), indicating the effectiveness of the DBN algorithm used in this paper.

In addition, Table 1 shows that the DBN classification results for flexion and extension movement involving the right and left arms are better than those for flexion and extension imagery involving the right and left arms. We infer that the HbO feature evoked by an executed movement may be more significant than that evoked by an imagined movement. It could also be that the signal-to-noise ratio for flexion and extension movement involving the right and left arms is greater than that for flexion and extension imagery involving the right and left arms. Secondly, Table 2 shows that the DBN classification result for a test set from one subject trained with the training set from the same subject is better than that of a test set trained with training set from different subjects, even while using the same DBN model. The fNIRS signal induced by this is different due to the difference in MI psychological activity between the subjects. It is necessary to construct and train a specific DBN classification model for each subject, that is, to construct a DBN model that varies from person to person. At the same time, the DBN model of a given subject can be promoted or migrated to other subjects' data within a certain classification accuracy, which can reduce the data collected from other subjects. For example, it is possible to apply a normal human DBN model to a disabled person.

Naseer et al. considered data extracted for different time windows between 20 s and 30 s after the start of the imagery task (starting time is 0 s) [29]. This is different from the time period for which data were extracted in this study.  Figure 5(b) shows that the average fNIRS response curve for flexion and extension imagery involving the right and left arms peaks at 16 s∼20 s. For online systems, the response delay in Naseer's study is limited by the conversion to online BCI. This study considers the conditional independence between RBM visible units [35]. We calculated, respectively, the correlation coefficients of L-HbO and R-HbO response curves for 0∼8 s and 8 s∼16 s in Figure 5(b): the correlation coefficient for 0∼8 s is 0.1231, and the correlation coefficient for 8∼16 s is 0.4509, indicating that HbO at 0∼8 s is more suitable as classification data.

In this study, we used the probability generation DBN model [34]. Since the optimal network topology is highly dependent on the type of problem and the distribution of training data, there is no general way to determine the number of layers and number of units in the hidden layer. Following from Hinton et al. combined with the number of training samples in this study, the number of units in the hidden layer [*h*_1_, *h*_2_] can be selected from 2 to 128, and it can be determined from the array [10, 20, 30, 40, 50] using the two-two cross-validation method. According to Lu et al. in the process of training DBN (the structure is 226 × 70 × 60 × 50 × 2), the number of samples in the training set needs to be greater than 100 to avoid overfitting [39]. In this study, the DBN structure used is smaller than the DBN structure adopted by Lu et al. To avoid overfitting, it is necessary to obtain a sufficiently large training set. Therefore, this paper takes the data of each sampling point as a sample. The training set is 19200 × 16 and the average training time is 5.17 s; the test set is 9600 × 16 and the average test time is 0.64 s. Compared to the study by Lu et al., even though the DBN has a small structure, the calculation speed is relatively faster and suitable for conversion to an online system.

Figure 5 shows an increase in HbO concentration and a decrease in HbR concentration during flexion and extension movement or imagery involving the left and right arms, which indirectly reflects an increase in neuronal population activity in the motor cortex [40]. Figure 5 also shows that the HbO concentration in the contralateral motor cortex is higher than the HbO concentration in the ipsilateral motor cortex during flexion and extension movement or imagery involving the left and right arms, indirectly indicating that the activation of neuronal population in the contralateral motor cortex is higher than that of the ipsilateral, which is consistent with existing research results [41–43]. Moreover, it can be seen from Figure 5 that the HbO amplitude during flexion and extension movement involving the left and right arms is higher than the HbO amplitude during flexion and extension imagery. This may be because actual movement activates more neuronal excitatory activity than MI, and the MI requires the subject to suppress actual movements.

### 4.1. Limitations and Outlook

The training set used in this paper has a low feature dimension of only 16 dimensions, which cannot be directly used in online systems. When converting to an online system, it is necessary to increase the feature dimension and reduce the sampling rate to avoid making the dimension of the input data too high and that of the training set too small to be fitted. Besides, due to the condition of experiment, we just recruited ten subjects which is relatively low. In the future, we will increase the number of subjects which may improve the classification accuracy and we will build an online MI-BCI system based on DBN and fNIRS, using online feedback to promote subjects to adjust their motor imagery mental activity strategy. This is expected to further improve the DBN classification performance.

For BCI applications, the inherent delay in the response of hemodynamics makes the generation of commands using fNIRS slower compared to EEG. A hybrid system approach, specifically the combination of fNIRS with EEG, may be useful to remove this kind of disadvantage [44]. Recently, the simultaneous measurement of fNIRS with EEG showed promising results [45]. In the future research, we will explore the hybrid fNIRS-EEG system to reduce the brain signal detection time or to increase the number of commands without sacrificing the classification accuracy.

## 5. Conclusions

In this study, a DBN algorithm based on RBM was constructed and used to classify fNIRS signals related to flexion and extension movement or imagery involving the left and right arms. The results show that the DBN algorithm can effectively identify flexion and extension imagery involving the left and right arms using fNIRS signals. In addition, it was shown that, for a given DBN model, better classification accuracy was achieved for the test dataset for a given subject when the DBN model is trained with training dataset from the same subject than when it is trained with a set from different subjects. This implies that a specific DBN model needs to be constructed and trained for each subject. However, the DBN model for one subject can be generalized or transferred to other subjects' data within a certain classification accuracy, which can reduce data collection from other subjects. It is expected that the study will lay a foundation for constructing online MI-BCI systems based on DBN and fNIRS.

## Figures and Tables

**Figure 1:** Experimental paradigm. (a) Timing of task prompts and task execution in a trial; (b) timing of a session.

**Figure 2:** (a) Schematic diagram of layout of the fNIRS signal acquisition probe (16 channels, 6 transmit probes, and 8 receive probes). Black rectangles indicate fNIRS source transmitter probes; black circles indicate fNIRS receiver probes, while black solid lines indicate fNIRS channels. (b) Experimental setup.

**Figure 3:** Schematic diagram of a single RBM model.

**Figure 4:** Schematic diagram of the DBN structure, *V* is the visible layer, *H* is the hidden layer, and the top is the output layer.

**Figure 5:** Average fNIRS response and topographic map. (a) The average fNIRS response of flexion and extension movement involving the right and left arms and topographic map of HbO concentration in the motor cortex during the first 8 seconds of performing the task. (b) Average fNIRS response for flexion and extension imagery involving the right and left arms and topographic map of HbO concentration in the motor cortex during the first 8 seconds of performing the task. In the figure, L-HbO and R-HbO are the *z* value of HbO concentration for flexion and extension movement or imagery involving the right and left arms; L-HbR and R-HbR are the *z* value of HbR concentration for flexion and extension movement or imagery involving the right and left arms; L-FE_ME: left arm flexion and extension execution; R-FE_ME: right arm flexion and extension execution; L-FE_MI: left arm flexion and extension imagery; R-FE_MI: right arm flexion and extension imagery.

**Table 1:** DBN classification accuracy for flexion and extension movement or imagery involving the left and right arms (%).

Subject number	Flexion and extension movement for right and left arms	Flexion and extension imagery for right and left arms
S1	86.90	81.79
S2	82.32	79.23
S3	81.47	70.94
S4	85.79	79.29
S5	76.23	73.97
S6	89.21	82.93
S7	84.79	78.56
S8	82.29	81.47
S9	78.04	73.96
S10	86.45	79.79
Mean	84.35 ± 3.86%	78.19 ± 3.73%

**Table 2:** DBN model classification results (%) for test dataset from one subject trained with training dataset from other subjects.

MODLE	(*h*_1_, *h*_2_)	S1	S2	S3	S4	S5	S6	S7	S8	S9	S10
DBN_S1	(10, 30)	**81.79**	78.97	80.43	76.89	78.52	76.87	78.69	80.06	68.79	78.93
DBN_S2	(10, 10)	77.92	**79.23**	76.27	75.06	77.92	75.97	77.67	74.26	75.31	69.93
DBN_S3	(10, 40)	68.71	66.17	**70.94**	67.46	68.71	64.93	66.56	64.48	63.26	64.43
DBN_S4	(10, 10)	79.25	77.49	76.85	**79.29**	75.43	79.25	77.49	71.85	77.29	69.25
DBN_S5	(10, 50)	72.06	68.16	72.79	71.93	**73.97**	69.06	61.69	69.79	69.93	66.06
DBN_S6	(10, 30)	79.56	77.43	76.87	78.25	76.32	**82.93**	79.23	67.26	66.76	79.31
DBN_S7	(10, 10)	73.56	76.43	76.87	68.93	69.32	77.64	**78.56**	69.26	71.97	73.67
DBN_S8	(10, 30)	77.06	76.83	75.97	76.43	76.12	75.34	75.56	**81.47**	76.67	77.67
DBN_S9	(10, 50)	64.26	65.31	72.93	67.13	69.48	70.26	60.43	71.76	**73.96**	70.77
DBN_S10	(10, 30)	75.96	77.23	69.45	77.9	65.87	74.12	75.94	76.87	76.98	**79.79**

DBN_S1, DBN_S2,…, DBN_S10, respectively, represent DBN models trained using training sets S1, S2,…, S10, and (*h*_1_, *h*_2_) are the number of units of two hidden layers of DBN.

## Data Availability

The data used to support the findings of this study are available from the corresponding author upon request.
